This article has been retracted.

# Prevention and Treatment of Sports Injuries and Rehabilitative Physical Training of Wushu Athletes

**DOI:** 10.1155/2022/2870385

**Published:** 2022-04-30

**Authors:** Shenghai Wu, Xin Luo

**Affiliations:** ^1^Sergeant College, Hunan Sports Vocational College, Changsha, 410000 Hunan, China; ^2^Sports Department, Hunan Sports Vocational College, Changsha, 410000 Hunan, China

## Abstract

This paper is aimed at exploring the characteristics of research on prevention and treatment of sports injuries and rehabilitation physical training of Wushu athletes. It also considers the application of rehabilitation physical training in the rehabilitation of Wushu athletes. By searching literature, conducting questionnaires, and combining mathematical statistics, it studies the injury prevention and rehabilitation training of Wushu athletes. This paper chooses the level of first class and above of sports, and a total of 50 elite male and female Wushu athletes were systematically trained as subjects of study. Athletes, aged 15 to 20 years, were trained for 2 to 5 years, 35 male athletes and 15 female athletes. Different from traditional rehabilitation therapy, athletes' physical rehabilitation training is also different from traditional sports rehabilitation treatment. By evaluating the physical condition of athletes, the causes of sports injuries were analyzed, to formulate special rehabilitation training programs and carry out athletes' rehabilitation training targeted and purposeful. Record the experimental data and analyze the experimental results. The experimental results show that physical rehabilitation training can make athletes avoid the influence of unsafe factors of sports injury, improve the safety of training, and effectively prevent sports injury. The experimental results show that physical rehabilitation training combined with rehabilitation medicine has obvious advantages, which can make Wushu athletes recover quickly without sequelae.

## 1. Introduction

Physical fitness is an important manifestation of athletes' athletic performance. The stress that the body can withstand and the limits of the body's ability to withstand the hit and the load of the body are based on daily training, which is the accumulation of daily training [1]. Because the strength and density of martial artists before the game is very high, the training is quite extensive and directs confrontation training. This kind of training can easily lead to fatigue. During the training, the mind is not concentrated, and some even continue to participate in the struggle during the disease stage [2]. However, strenuous exercise is more likely to cause new sports injuries or worsen the original damage. In addition, due to intensive training, the load on some parts of the body is too large; so, these parts are easily damaged. If a martial arts athlete receives special technical training, he must first practice the technique and then perform special strength training with his hand and waist. When training legs, etc., the load is relatively intensely concentrated on the elbows, waist, and knees, which can also cause fatigue and damage in various parts [3]. New rehabilitation training can improve your health and meet your daily exercise needs. Physical rehabilitation training is a comprehensive discipline that helps to correct and restore motor dysfunction using physical training methods, also known as rehabilitation training [4, 5]. Physical rehabilitation training is different from traditional sports training. It has a strong correlation and help and is a new concept of sports training. In sports, the athlete's physical performance (including general physical fitness and physical fitness) is the basis of the athlete's athletic ability [6, 7]. At present, the physical fitness of Chinese athletes is mostly in a state of poor health. As part of special sports training, athletes are subject to various injuries or injuries. Traditional medical rehabilitation methods cannot quickly solve the problem of athlete training. Physical rehabilitation training can better promote the recovery of athletes' physical fitness and improve their physical fitness. Physical rehabilitation training effectively combines various concepts such as sports medicine, functional rehabilitation, exercise training, and sports nutrition [8, 9]. The causes of athletes' sports injuries and the use of personalized rehabilitation training methods and nutritional supplements to improve athletes' health effectively prevent sports injuries and enable athletes' physical function and physical health to meet specific exercise requirements [10, 11].

Long-term large-scale exercise training makes the athlete's muscle strength unbalanced, resulting in decreased joint stability or joint displacement, resulting in joint damage in athletes during daily training. This requires effective training methods to prevent the occurrence of sports injuries and help athletes to recover quickly. In sports training, no matter how serious the sports injury, the athlete's physical fitness will decline, and the decline in physical fitness will aggravate the injury. Therefore, when there is a sports injury, only medical rehabilitation cannot completely treat the injury of the athlete [12, 13]. Physical rehabilitation training combines rehabilitation and physical training. It can carry out physical exercise while the athlete performs rehabilitation training, promote the recovery of the athlete's physical health, and make the athlete's physical state transition to the best state, which not only meets the needs of sports training, uninterrupted, shortening the athlete's physical recovery time and providing a strong guarantee for the athletes to resume normal training [14, 15]. Physical rehabilitation training includes rehabilitation. Unlike traditional exercise rehabilitation therapy, it evaluates the athlete's physical condition from both nutritional support and sports medicine, analyzes the causes of sports injuries, and develops special rehabilitation training programs based on the athlete's injury. Targeted and purposeful athlete rehabilitation training is as follows: physical rehabilitation training can enable athletes to avoid the unsafe factors of sports injuries, improve the safety of training, and effectively prevent the occurrence of sports injuries [16]. At the same time, during the athlete's physical exercise, the corresponding training can be used to treat the athlete's injury, promote the athlete's health recovery, and shorten the treatment time [13, 17].

This paper applies the research findings of the scholars. Scholars such as Shutze contacted eligible patients by phone and invited them to complete nine surveys to assess the long-term effects of FRR. The use of analgesics, postoperative physical therapy time, patient satisfaction, symptom relief, activities of daily living, athletic performance, exercise recovery time, etc. is as follows: multivariate analysis of risk factors: age, chest muscle release, preoperative anesthesia use, and exercise load. takes part in throwing exercises. Results are as follows: 232 athletes met the inclusion criteria, of which 67 (14-48 years; 35; 99% were white) answered the survey. The average time from surgery to investigation was 3.3 years (2.2-7.0 years). The most common sports in this group are baseball and softball (*n* = 44 [66%]), volleyball (*n* = 7 [10%]), cheerleaders, and gymnastics (*n* = 5 [7%]), from high school to professional level [14]. The results of the survey showed that 96% of painkillers improved, 75% required contralateral FRRs, 82% had symptomatic regression, 94% had unrestricted daily activities, and after FRRs, 70% returned to the same or better exercise level which reached 50% during the year. Multiple regression analysis found that the younger the age, the more predictable the duration of physical therapy. Conclusion is as follows: in this center, 40% of patients who require FRR treatment are competitive athletes. The results of this study show that most companies are able to return to precompetitive status after FRR, and there is almost no empirical limit in daily activities. Within six months of surgery, half of the game can return to pr-disease levels. Most people are satisfied with the decision to accept the FRR. Further research is needed to determine the predictors of successful recovery of competitive sports [15, 16]. Hoover and other scholars have found that as strength and training coaches increasingly use phased models to inform athletes about their training programs, athletes' exercise prescriptions and training programs are growing rapidly. Similarly, exercise prescriptions and exercise processes are the basic skills of a sports therapist and are necessary to balance the physical stress of injury and recovery of the athlete [17, 18]. This course will outline the staging model of a sports therapist and its application in rehabilitation. They found that models of exercise prescriptions and exercise progression were developed both in theory and scope, and that these models helped to improve the resilience of countless athletes compared to the care of previous generations of athletes. Despite this, despite these advances, these models often do not fully bridge the gap between these rehabilitation programs and coaches to help athletes reach their peak. More staging model knowledge can help sports therapists assess, clinical reasoning skills, exercise progression, and goal setting, enabling athletes to continue to participate in high-level competitions [19, 20].

Different from the traditional sports rehabilitation treatment, the injury situation and physical rehabilitation training of athletes are different from traditional sports rehabilitation therapy. They evaluate the physical condition of athletes, analyze the causes of sports injuries [21, 22], and analyze the causes of sports injuries. The situation is formulated with a special rehabilitation training program to carry out rehabilitation training for athletes in a targeted and purposeful manner [23].

## 2. Proposed Method

### 2.1. Body Shape Characteristics of Martial Arts Mobilization

Martial arts are classified according to the dominant factors of competitiveness and belong to the difficulty performance of skills; according to the classification of action structure, they belong to variable combination items in multiaction structure. The physique characteristics of martial arts routine athletes are usually body shape, facial features, slightly longer neck, shorter clavicle and scapula, slightly longer limbs, straighter arms, longer calves than thighs, straight knees, slightly shorter ankles, and thinner Achilles tendons. Clear, hands and feet are large, the pelvis is narrow, the buttocks muscles are tightened upwards, and the muscles are peeled off. From a physical function point of view, technology-led athletes, if aesthetically difficult to please, need good cardiovascular, nervous, and visual, auditory, and other sensory system functions.

### 2.2. Operational Requirements

In order to develop martial arts as part of competitive sports, we must move in this direction. This is the development model of the world's hard and beautiful sports and also the requirements of the competitive sports technology movement. If the technical characteristics of competitive martial arts form the essence of competitive martial arts, then “high, difficult, beautiful, new, stable” is the requirement of martial arts training. During the drilling process, the attitude, direction, and force of the action are required to achieve the standardization of the action, the accuracy of the method, the graceful shape, and the grounding action.

### 2.3. Training Requirements

Martial arts is a high-intensity, short-term intermittent exercise. Its functional mode is based primarily on the aerobic and anaerobic threshold characteristics of lactic acid. In order to improve the endurance of martial arts athletes in competitions, aerobic and anaerobic training is needed to improve their endurance and ability. Athletes have high physical fitness and pay special attention to the function of lactic acid anaerobic training. Therefore, strength, speed, and endurance are essential for excellent martial arts athletes, and all three are indispensable. Prematch training due to different levels, different strengths, different opponents, etc., the damage caused in actual combat, it is likely to cause acute injury due to the use of weight difference, directional error, and excessive technical action. In the investigation, the knee joint was the most damaged, because the martial arts movement could not do without the knee joint strength from standing to squatting. In order to participate in a level that is more conducive to their excellent performance, martial arts athletes need to strictly control their weight in pre-competition training, but because they do not reduce the amount of exercise, even in the process of controlling weight, increase the amount of exercise, exercise load increases, due to weight. The excess water and fat are reduced, the water cannot be replenished after training, the body's water cannot reach equilibrium, the muscle loses its original elasticity, and the stretch of the ligament is also reduced. Because fat protects the body and joints, joint loss is lost if fat is reduced. Therefore, athletes control their weight with large capacity and high intensity before the game, which is prone to sudden damage. Before the game, the athletes were physically exhausted and their ability to each part decreased. It tends to be listless, with nerves and muscles sticking stronger than usual, especially for athletes who control their weight before the game. Ordinary people must be strong. General preparation activities can reach the central nervous system excitement in 15 minutes, while weight control athletes need 18 to 35 minutes or even longer. Therefore, if the athlete neglects the preparatory activities before training and performs heavy-duty and high-intensity exercises, it is easy to cause sports injuries.

### 2.4. Training Guidance

The so-called training guiding ideology refers to the theoretical understanding of the characteristics of sports, the actual situation of sports teams and athletes, and the expected goals achieved through training practice. According to the guiding ideology of the characteristics of competitive martial arts, the martial arts training program aims at the development trend of “beauty, high, new and stable,” using a large amount of theoretical knowledge, combined with sports practice, and training according to the principles of the system. Sports training examples, sports training and technical principles combined with sports characteristics, strength, and endurance training are the core principles of training. Unreasonable technical actions cause damage. Athletes cannot master the technical and technical essentials scientifically and correctly, and it is very easy to cause damage during training. This puts higher demands on the martial arts coaches, not only asking the coaches to teach the athletes technical movements but also asking for teaching.

The trainer explains the principle of technical movements and explains the principles that help athletes to use their brains to find ways to attack their opponents and how to restrain their opponents' attacks, without being damaged during training.

### 2.5. Training Content

Martial arts have a more comprehensive physical fitness requirement for athletes. According to the characteristics of martial arts and the needs of technological development, martial arts athletes should focus on speed, strength, jumping ability, flexibility, agility, and endurance training. Martial arts athletes must practice hands, eyes, body, step, spirit, qi, force, and these movements in the field and always support strong physical strength. Traditional basic martial arts skills and basic sports practice are important tools for developing martial arts' special physique. The martial arts athlete's body not only can get a more comprehensive exercise but also can improve the flexibility and coordination of each joint, improve the control of muscle flexibility and improve the function of the body-related structure. On the other hand, the level of equipment upgrade technology also laid the foundation for athletes. Stretching in combat, the goal of stretching soft tissue and muscle in martial arts is to be more flexible in exercise, stretching soft woven or relaxing muscles during exercise, which helps to eliminate muscle fatigue and maintain muscle elasticity. Prevent muscle tension and avoid deformation and stiffness of sports equipment. Stretching exercises are mainly used to prepare and the final action. The main purpose of active stretching is to minimize the internal viscosity of soft tissues and muscles before training, to keep it light, to increase muscle temperature, increase elasticity, and to prevent muscle tension during training, thus requiring active stretching. In addition, the main purpose of stretching after exercise is to relax the muscles after exercise, to get rid of fatigue, accelerate the release of muscle metabolites, reduce muscle soreness, and allow athletes to restore their body shape as soon as possible, ready for the next muscle exercise. The method of stretching after training mainly uses passive stretching, allowing athletes to stretch each other or let the trainer stretch.

### 2.6. Sports Training Methods and Methods for Athletes

#### 2.6.1. Strength Training

Martial arts is a combination of exercise and rest, with a focus on “lightning movement.” In martial arts, the difficulty of jumping and the difficulty of balancing static movements both require static muscle strength. In general, fitness training, speed, and strength training should be performed first. For loads, athletes use a maximum load of 40% to 600 and perform 6-8 sets. In order to increase maximum strength, athletes weigh from 100% to 120%, barbells, semicircles, jerk weights, etc., as well as 4-6 groups, intermittent training methods and repeat methods. Finally, in the development of strength endurance, strength endurance should be the main content of strength training, and you can use about 80% of the maximum strength for strength training until the body is exhausted; in the process, you can use some training tools group cycle. Special strength training uses martial arts in the form of bows, “horse,” or “equestrian” steps, steps, virtual steps, steps, etc. These basic achievement methods can improve the static strength of martial arts. In addition, martial arts athletes also need good motivation and mainly use super-sensory, jumping, flashing, display, ripple, spin, fold, and other personal practice skills.

#### 2.6.2. Speed of Quality Training

Movement speed is the core of completing martial arts. Only “a fist - like a meteor, the eyes are like electricity”. For routine training, athletes must demonstrate the characteristics and style of wavy, fast, bold, and enduring martial arts. In addition, athletes must complete many actions in a short period of time.

#### 2.6.3. Flexible Exercise

Flexible, high-quality martial arts exercises use artificial methods such as vibration, displacement, stretching, and torsion to stimulate the external forces of the shoulders, arms, waist, legs, and ankles to obtain joints, muscles, tendons, and ligaments. Develop the flexibility of the above components. Basic skills in basic and basic sports can enhance athletes' flexibility. Such as shoulders, shoulder pressure training, ring, arm, and other exercises, the legs have positive pressure, the legs have side pressure, the hind legs are pressed, the legs have a positive pulling force, the legs have a back, the legs are pushed, and the legs are kicked.

#### 2.6.4. Other Physical Health

In addition to good strength, speed, and flexibility, martial arts athletes must have good quality endurance, sensitivity, and coordination. As for endurance, you can run 400-800 meters quickly and use the overtime training method, that is, do half or two trainings without interruption, to improve the athlete's endurance in sensitivity and coordination. It can be improved through special training, such as improving knee balance, swallowing balance, and exercising with the ball.

## 3. Experiments

### 3.1. Experimental Settings

#### 3.1.1. Research Object

This paper selects the level 1 and above sports level and 50 male and female excellent martial arts athletes who are systematically trained as the research object. The athletes are 15 to 20 years old, with a training period of 2-5 years, 35 male athletes and 15 female athletes. Different from the traditional sports rehabilitation treatment, the injury situation and physical rehabilitation training of athletes are different from traditional sports rehabilitation therapy. They evaluate the physical condition of athletes, analyze the causes of sports injuries, and analyze the causes of sports injuries. The situation is formulated with a special rehabilitation training program to carry out rehabilitation training for athletes in a targeted and purposeful manner. Physical rehabilitation training mainly includes three types: the first type of physical fitness athletes to improve their physical fitness and athletic ability; the second type of athletes in the injured or subhealth state to diagnose the athlete's physical condition, find out the reasons for the decline in physical fitness, and develop special training to restore the athlete's health; the third category through specific physical fitness training to help athletes reduce the pain and restore exercise capacity.

#### 3.1.2. The Experimental Arrangement

In this experiment, 50 Wushu athletes were trained in three stages for 6 weeks.

### 3.2. Functional Rehabilitation Physical Training

For various reasons, the athlete's physical fitness will decline after the injury, and the decline in physical fitness will reduce the athlete's own recovery ability and increase the athlete's injury. Therefore, once an athlete is subjected to sports injuries, in order to ensure that his athletic ability and function are not harmed, it is necessary to combine the relevant knowledge of rehabilitation medicine with the function and institutional needs of the physical activity to recover, according to the actual situation of the athletes bodies, and the relevant knowledge of rehabilitation medicine is the fulcrum. Stand up for skill-based rehabilitation physical training, timely adjust the rehabilitation program according to the problems existing in the rehabilitation physical training, and promote the early rehabilitation of athletes' injuries.

### 3.3. Physical Training for Disease Prevention and Rehabilitation

Athletes often need to exercise for a long time, which can lead to muscle fatigue or joint instability, which can easily cause different degrees of damage. Effective prevention of physical injuries is very important for physical education. By analyzing the damage mechanism, an appropriate training plan is developed, and measures are taken to avoid damage in practice to effectively prevent the deterioration of injured athletes and avoid repeated injuries. For example, humeral pain is one of the common injuries of athletes, mainly due to the imbalance of muscle strength inside and outside the thigh, resulting in displacement of the lower leg. If the knee is stretched during training, this will exacerbate the pain caused by abnormal movement of the lower leg. Therefore, during sports, avoid injury to the athlete's sports injuries; so, a closed-circuit exercise with a fixed foot position should be chosen to position the knee and toe vertically to relieve pain and avoid knee flexion.

### 3.4. Functional Rehabilitation Physical Training

Functional rehabilitation training is an important principle of physical rehabilitation training. In sports training, most of the movements are three-dimensional movements performed by multiple joints. A drop in joint function can cause the movement to fail or fail to meet the standard. For example, in a baseball throw, the abdominal muscles simultaneously participate in abdominal adduction and rotation. The traditional sit-up training does not aim at the training of the abdominal muscles and cannot fully exert the advantages of coordinated movements such as the abdomen, lumbar vertebrae, and upper limbs. If we use the rubber band tension to do the sit-up abdominal abdomen adduction exercise, we can better exercise the abdominal muscle function and make the athlete more flexible.

### 3.5. Neurological Rehabilitation Physical Training

The center of the body is an important part of maintaining body posture and ensuring body movement. In traditional sports training, there is no exercise or pertinence for the center of the body. More than half of the central muscles of the trunk are vertically or horizontally aligned. Traditional sit-ups are not enough to exercise nerves. Refined abdominal flexion and rotation in physical rehabilitation training can fully exercise the central muscles of the trunk, stimulate the central nervous system, and better coordinate the posture and movement.

### 3.6. Balance and Joint Rehabilitation Physical Training

Balance and joint stability training is the primary method of preventing joint damage. Balance training in physical rehabilitation, simple equipment is often used to achieve the required exercise requirements. For example, trampoline athletes often sprain their ankles. During training, they usually use a balance board to balance their ankles. After a month or so of training, the ankle joint muscle group is significantly enhanced, and it is easy to complete the balance control of the unstable plane and improve the athlete's balance control ability: the function of the joints.

## 4. Discussion

### 4.1. Functional Rehabilitation Physical Training

When an athlete is injured, first assess the degree of injury, consult relevant medical books, and develop their functional rehabilitation physical training. Three sets of experiments were set up, as shown in Table 1. For example, each group of 15 male athletes suffered an ankle injury. The external application of Yunnan white ointment was taken, and the western medicine was taken orally. The training continued except for the ankle. The training intensity and ankle recovery of the athletes are shown in Table 2. After fully recovering from the athletes, the proficiency of the original action is shown in Table 3.

Table 2 shows that the longer the training time, the longer the recovery time is consumed.

Table 3 shows that the longer the training, the higher the proficiency of the original movement.

### 4.2. Disease Prevention Rehabilitation Physical Training

Athletes usually need long-term exercise training, which can cause muscle fatigue or joint instability, which can easily cause different degrees of injury. Effective prevention of injuries in physical training is essential for sports training. By analyzing the mechanism of injury, formulating relevant training programs, and choosing to avoid the movements that cause athletes to hurt, practice to effectively prevent the injury of the injured athletes and avoid the occurrence of reinjury. The experiment analyzed the impact of the relevant actions on the related injuries with the recovery time as a reference, as shown in Figure 1.

Figure 1 shows that the ankle is prone to injury when flipping, and the knee is prone to injury when bouncing.

### 4.3. Functional Rehabilitation Physical Training

In the long term, a large number of sports training, the muscle strength of athletes is not balanced, which leads to a decrease in joint stability or joint displacement, which leads to joint injuries in athletes during daily training. In the case of sports injuries, athletes must influence their physical fitness and cannot perform various training sessions or compete. It also requires effective training methods to prevent sports injuries and help athletes recover as soon as possible. In sports training, no matter how serious the injury, this will lead to a decrease in the athlete's physical strength, and a decrease in physical fitness will aggravate the injury. Therefore, when there is a sports injury, only medical rehabilitation cannot fully treat an athlete's injury. Physical rehabilitation combines both rehabilitation and physical preparation, and it can perform physical training of athletes during rehabilitation, help restore athletes' physical fitness, and ensure that the athlete's physical condition is in a better condition, which not only corresponds to sports training. Continuous, it reduces the athlete's physical recovery time and provides a reliable guarantee of a special training after the athlete returns to normal. Physical rehabilitation training includes rehabilitation therapy; unlike traditional sports rehabilitation therapy, it assesses the physical condition of athletes in terms of nutrition support and sports medicine, analyzes the causes of sports injuries, and develops special rehabilitation training programs in accordance with the injuries of athletes. Physical rehabilitation can help athletes avoid unsafe factors that cause sports injuries, improve training safety, and effectively prevent sports injuries. At the same time, during the physical preparation of athletes, appropriate training can be used to treat injuries to athletes, to help restore athletes' health, and reduce treatment time. A decrease in joint function can result in incomplete or inconsistent exercise, attempting to adopt a new action or training method, randomly grouping 25 groups of each group, and the questionnaire is satisfied with the current action and the improvement of future actions. The attitude is shown in Figures 2 and 3. A questionnaire for the number of people looking forward to improvement and having a good method is shown in Figure 4 for each age group.

Figure 2 shows the highest satisfaction with jumps and the lowest satisfaction with spins.

Figure 3 shows the highest percentage of positive optimism, while the percentage of full and partial changes is the same.

### 4.4. An Important Part of an Athlete's Athletic Ability Is Physical Health

There is an important manifestation of sports skills in daily training of athletes practice. The development of medical technology to this day, the practice of physical rehabilitation, and this new teaching method has been widely used in sports training. Physical rehabilitation can effectively help athletes to restore health and control healing injuries and prevent recurrence, and improve fitness to meet the needs of daily training. In the training, there are deep understandings of the athletes of various movements, and the number of people who are looking forward to improvement and good methods is 10 in each age group as shown in Figure 4.

Figure 4 shows that people aged 18-23 are more expected to improve.

## 5. Conclusions

1. During the experiment, it was found that the human muscles were divided into large muscle groups and small muscle groups in the form of fixed joints. General strength exercises are usually performed on large muscle groups, ignoring the practice of small muscle groups. The damage caused by the battle is difficult to deal with, and many harmful upper limb exercises are needed to recover. Conversely, training a small group of muscles with a small weight of rubber tension band or small dumbbells can be more easily trained and does not allow injury. In addition, small muscle groups typically have multiple directional motor functions and are also multidirectional in training. Small muscle groups move more accurately than large muscle groups, and they can be easily trained in place, which puts high demands on the trainer's biomechanics and human anatomy
2. Joint stability and balance training can effectively prevent joint damage. Since joint stability is mainly determined by joint body sensation, joint body sensation plays an important role in time. Adjusting the position of the joint and preventing damage, balance training usually uses unstable plans to restore and utilize the power of proprioception. In foreign balance training courses, balance equipment of various difficulty levels is designed using simple equipment such as ski balance, hemisphere, fitness ball, and balance board. Take martial arts as an example: he usually has an ankle sprain, and his limbs cannot be properly trained without the thick bandage. Therefore, we require athletes to use the balance board to balance the ankle joints. At first, the athlete can complete the training in 2-3 seconds. But after a month of balanced training, the muscles around the ankles will strengthen and stand for more than 5 minutes without falling. The result is that athletes no longer need a lumbar support ankle and can return to the team for normal exercise. Martial arts exercises involve stretching soft tissues and muscles before, during, and after struggling, so that stretched soft tissue or muscles are completely relaxed. This helps to eliminate muscle fatigue, maintain muscle elasticity, prevent muscle tension, and prevent technical deformation and stiffness. Stretching is primarily used to prepare and organize activities. The main goal of stretching is to minimize the internal viscosity of soft tissues and muscles before training, increase muscle temperature and elasticity, and prevent muscle damage during training. Use active stretching exercises. The main purpose of stretching after exercise is to relax the tense and tired muscles after exercise, accelerate the release of muscle metabolites, relieve muscle irritation, and allow athletes to restore their body shape as soon as possible, in preparation for the next exercise
3. Through the analysis and comparison of the data, it is found that the injury and physical rehabilitation training of athletes in daily training is different from traditional sports rehabilitation therapy, starting from the support of nutrition and sports medicine, by assessing physical fitness, athletes' condition, and sports injuries. The reason for this is that a special rehabilitation training program was developed based on the athlete's traumatic situation, and the athletes were purposefully and purposefully trained for rehabilitation. The experimental results show that physical rehabilitation training can enable athletes to avoid the unsafe factors that cause sports injuries, increase the safety of training, and effectively prevent the occurrence of sports injuries

## Figures and Tables

**Figure 1:** Related actions on the impact of related injuries.

**Figure 2:** Satisfaction with the current action.

**Figure 3:** Attitudes toward future action improvement (%).

**Figure 4:** Looking forward to improvement and good methods.

**Table:** (a) Knee rehabilitation training

Training goal	Training methods	Time/times	Group number
Knee stability training	Lunge stability exercises	1 min	5
The first stage	One-legged, closed-eye combat	1 min	3
	Quiet squat down against the wall	1 min	3
	Rubber band lunges	30s	5
	Kettlebells pull hard on one leg	15 times	1
Lower limb stability training	Rubber band lunges	1 min	3
The second stage	A suspended one-leg lunge squat	20 times	3
	Lie on your back a hip	1 min	3
	The belly bridge is supported at four points	1 min	3
	Side of the bridge	40s	3
Lower limb strength enhancement	Assist with one-leg squats	10 times	3
The third stage	Lunge stability exercises	1 min	5
	Stand on one leg with eyes closed	30s	3
	Abutment bridge 4 or 3 point support	30s	3
	Side of the bridge	1 min	3

**Table:** (b) Ankle rehabilitation training

Functional ankle exercises	Plantar and calf fascia combing	30 s for each part	2
The first stage	Minibelt stretching exercises	15 times	3
	Minibelt inside and out exercises	15 times	3
	Squat ankle joint flexion and extension, inside and outside the exercise	15 times	3
	Heel raises during the march	15 times	3
	Supine crunches	12 times	3
	Lie on your back with scissors legs	12 times	3
Ankle stability exercises	Plantar and calf fascia combing	30 s for each part	2
The second stage	Soft pad 1/4 shallow squat exercises	15 times	3
	Soft pad 1/4 single side shallow squat exercises	8 times	3
	Wave speed ball squats	15 times	3
	Wave speed ball switch foot single side squat exercises	8 times	3
Ankle strength exercises	Plantar and calf fascia combing	30 s for each part	2
The third stage	Dumbbells squat on one side	8 times	3
	Wave speed ball dumbbell squat on one side	8 times	3
	During the march dumbbell up lunge	8 times	3
	Unilateral rhea stability training + one foot jump on cushion training	8 times	3
	Drop the medicine ball in the kneeling position	8 times	3
	Drop the medicine ball on your knees. - sideways	8 times	3

**Table 2:** Training intensity and ankle recovery.

	3-5 days recovery	5-10 days recovery	10-15 days recovery
Training for 2 hours	10	5	0
Training for 5 hours	5	7	3
Training for 8 hours	3	4	8

**Table 3:** Proficiency of the original action (%).

	0-50	50-80	80-100
Training for 2 hours	9	6	0
Training for 5 hours	6	7	2
Training for 8 hours	3	5	7

## Data Availability

The data that support the findings of this study are available from the corresponding author upon reasonable request.
